The article "In Vitro Antimitotic and Hypoglycemic Effect Study and Acute Toxicity Assessment of the Aqueous and Organic Extracts of Chamaerops humilis L. var. argentea Andre" was published in 2022. Journal: Biomed Res Int.

# *In Vitro* Antimitotic and Hypoglycemic Effect Study and Acute Toxicity Assessment of the Aqueous and Organic Extracts of *Chamaerops humilis* L. var. argentea Andre

**DOI:** 10.1155/2022/4303506

**Published:** 2022-10-14

**Authors:** Nacima Lachkar, Fatima Lamchouri, Hamid Toufik

**Affiliations:** Laboratory of Natural Substances, Pharmacology, Environment, Modeling, Health & Quality of Life (SNAMOPEQ), Polydisciplinary Faculty of Taza (FPT), Sidi Mohamed Ben Abdellah University (USMBA) of Fez, B.P.: 1223 Taza-Gare, Taza, Morocco

## Abstract

*Background. Chamaerops humilis* L. var. argentea Andre is a plant widely spread in the region of Taza (North-East of Morocco); it is used in traditional phytotherapy against cancer, diabetes, inflammations, cardiovascular and respiratory diseases, and for the treatment of digestive disorders. *Objective and Methods.* The objective of our work is to contribute firstly, to the study of the *in vitro* antimitotic potential by the phytotest of *Lepidium sativum* and the evaluation of the *in vitro* antidiabetic activity of three enzymes (*α*-amylase, *α*-glucosidase, and *β*-galactosidase) on nine aqueous and organic extracts prepared from the leaves of *Chamaerops humilis*. In addition, a correlation study was carried out on the chemical composition and the antimitotic and antidiabetic activities of *Chamaerops humilis* leaves. Then, we tested the acute toxicity of the decocted extract and the ethanolic extract. *Results.* The results of the antimitotic activity showed that the decocted extract showed a higher inhibitory activity than the other aqueous extracts (IC_50_ = 9.624 × 10^3^ ± 95.97 *μ*g/mL); for the organic extracts, the ethanolic extract and ethanolic macerated expressed the highest values for the cell growth inhibition test with an IC_50_ of 5.638 × 10^3^ ± 22.61 and 5.599 × 10^3^ ± 45.51 *μ*g/mL with statistically nonsignificant difference. Regarding the antidiabetic activity, the decocted showed a higher inhibitory activity than the other aqueous extracts for *α*-amylase (IC_50_ = 1.781 · 10^5^ ± 358.30 *μ*g/mL), *α*-glucosidase (2.540 × 10^2^ ± 3.14 *μ*g/mL), and *β*-galactosidase (7.118 × 10^2^ ± 16.13 *μ*g/mL); the ethanolic extract also revealed the highest inhibitory activity for *α*-amylase (IC_50_ = 8.902 × 10^3^ ± 57.81 *μ*g/mL), *α*-glucosidase (2.216 × 10^2^ ± 1.39 *μ*g/mL), and *β*-galactosidase (2.003 × 10^2^ ± 7.41 *μ*g/mL). A strong correlation was recorded between the antimitic activity and the inhibitory capacity of *β*-galactosidase and between these two activities and the chemical composition of *Chamaerops humilis* leaves. The acute toxicity study showed that the decocted and the ethanolic extract are weakly toxic with an LD_50_ greater than or equal to 5000 mg/kg. *Conclusion*. *Chamaerops humilis* could become a good source in traditional herbal medicine.

## 1. Introduction

The cancer represents one of the major causes of death in the world. In 2020, cancer was responsible for 10 million deaths worldwide [1]. In Morocco, tumors are the 2nd cause of mortality with a percentage of 13.4% of deaths, after the cardiovascular diseases [2].

Chemotherapy is an important treatment modality in oncology alongside other treatments [3]; however, the major problem with chemotherapy is that it is a nonspecific therapy; chemotherapeutic agents attack both the cancerous cells of the tumor and normal healthy cells, which can lead to multiple disorders in different organs; chemotherapy treatment leads to numerous changes in cell structure and function, resulting in progressive, continuous and often irreversible toxic side effects. In addition, chemotherapy is associated with various side effects, including cardiocytotoxicity, nephrotoxicity, myelosuppression, neurotoxicity, hepatotoxicity, gastrointestinal toxicity, mucositis, and alopecia, which severely affect the quality of life of patients with cancer [4]. Therefore, it is essential to carry out experimental research to find new anticancer agents that are more effective and less harmful.

Diabetes in its turn constitutes a real public health problem on a worldwide scale. In 2021, diabetes was responsible for 6.7 million deaths worldwide with 1 death every 5 seconds and 796.000 deaths in the Middle East and North Africa [5]. In Morocco, this disease causes more than 24.000 deaths per year [6]. Diabetes can cause multiple complications that require follow-up by health professionals, and this makes its management costly in terms of the expenses required to care for the diabetic person.

In fact, there is a strong association between cancer and diabetes; people with diabetes have a high risk of developing cancer. Indeed, numerous studies have demonstrated the relationship between diabetes and the occurrence of cancer. Diabetes and insulin resistance could be the consequence of an early, undiagnosed cancer, but, in addition, diabetes could also be related to the precancerous state of the pancreas that affects its insulin-secreting capacity [7]. Insulin resistance and its associated inflammatory disturbances also contribute to the carcinogenic potential of NASH (nonalcoholic steatohepatitis). In addition, it has been shown that for every 1 mmol/l increase in blood glucose, and there is a 10-20% increase in cancer risk (incidence/mortality) in men and women [8]. Indeed, in noninsulin-dependent diabetes, there is insulin sensitivity, which leads to hyperinsulinism and elevated circulating levels of insulin-like growth factors (IGFs) that are capable of stimulating cell proliferation in many organs, in particular the liver, pancreas, colon, ovary, and breast [7, 9, 10]. In addition, cancer is among the major causes of death in type 2 diabetes [11, 12].

Faced with this situation, the treatment of cancer and diabetes in Morocco is based mainly on the use of modern protocols and drugs, which can be costly for poor people who find it difficult to access modern health care. In this regard, traditional phytotherapy is widely used due to its availability and accessibility for the treatment of several pathologies [13–15].

Moroccan flora constitutes a real resource of natural molecules because of its richness and phytodiversity, which classifies Morocco among the countries that have a long medical tradition and traditional know-how based on medicinal plants [16]. For its part, the region of Taza (North Eastern Morocco) is distinguished by the diversity and richness of its natural environment and has one of the main and oldest national parks in Morocco, the Tazekka Park, which is characterized by a diverse natural abundance of aromatic and medicinal plants [17, 18]. Among these plants we mention, *Chamaerops humilis* L. var. argentea Andre is widely distributed and used by the local population in basketry for the manufacture of the doum basket, the palm heart is consumed as a seasonal fruit, and the leaves are used to feed the livestock [15, 18]. C. *humilis* is also used in traditional medicine to treat various pathologies including cancer [15, 19, 20] and diabetes [15, 21–24] and for the treatment of digestive disorders [15, 19]. Additionally, *Chamaerops humilis* is naturally abundant in the chemical compounds including gallic tannins, steroids and terponoids, saponins, and reducing sugars [19]. Furthermore, according to a mineralogical and phythochemical study that we have recently conducted [15], the leaves of *Chamaerops humilis* L. var. argentea are rich in minerals such as iron (82395.00 mg kg^−1^), potassium (9354.90 mg kg^−1^), phosphorus (1828.62 mg kg^−1^), magnesium (1312.47 mg kg^−1^), sodium (627.03 mg kg^−1^), copper (542.64 mg kg^−1^), calcium (92.19 mg kg^−1^), zinc (66.15 mg kg^−1^), and selenium and strontium (3.00 mg kg^−1^). In addition, the aqueous and organic extracts of this part of the plant contains catechic tannins, flavonoids, saponins, sterols, and free quinones. In addition, the aqueous and organic extracts of this part of the plant contains catechic tannins, flavonoids, saponins, sterols, and free quinones. The quantitative study also revealed that the aqueous and organic extracts of the leaves of *Chamaerops humilis* have high contents of phenolic compounds; the ethanolic extract and the ethanolic macerated have the highest values of total polyphenols, respectively, 96.99 ± 0.82 and 100.27 ± 1.95 mg EAG/gE, catechic tannins, respectively, 50.27 ± 0.99 and 52.11 ± 1.02 mg EC/gE with a statistically nonsignificant difference between these two extracts.

In Morocco, the strong progression of phytotherapy in recent years can pose risks for the consumers. Indeed, we have noticed that countless products and recipes based on plants or mixtures of plants are marketed on social networks and internet sites by unqualified people, which raises questions about the dose contained in these products and its conditions of extraction, manufacture, conservation, and possible interactions between the constituents of the product mixture or traditional recipe used. Ignorance of the use of medicinal plants can result in financial and human costs that will affect the national economy through the harmful toxic effects of the plants used [25, 26].

In view of these findings and as a continuation of the work carried out on *Chamaerops humilis* L. var. argentea Andre [15, 18], in the present work, we are interested in pursuing the validation of the therapeutic use of dwarf palm in traditional medicine through the *in vitro* study of its antimitotic and antihyperglycemic potentials of aqueous and organic extracts and the evaluation of its acute oral toxicity.

## 2. Material and Methods

### 2.1. Chemicals and Reagents

Colchicine, *α*-amylase from *Aspergillus oryzae*, starch, sodium phosphate buffer, dinitrosalicylic acid (DNS), acarbose, 4-p-nitrophenyl-*α*-D-glucopyranoside (pNPG), sodium carbonate (Na_2_CO_3_), *α*-glucosidase from *Saccharomyces cerevisiae*, *β*-galactosidase from *Escherichia coli*, 2-nitrophenyl *β*-D-galactopyranoside, quercetin, ethanol, chloroform, n-hexane, and dimethyl sulfoxide (DMSO) were used. These chemicals were purchased from Sigma Aldrich (Saint Louis, Missouri, USA).

### 2.2. Plant Material

The leaves of *Chamaerops humilis* L. var. argentea Andre used in the present study were collected in February 2017, in Bab Boudir located at 46 km from the city of Taza (Figure 1). The identification of the plant was carried out by Dr. Abdelmajid Khabbach, a reference sample “SB2017” was deposited in the herbarium of the laboratory Natural Substances, Pharmacology, Environment, Modelling, Health and Quality of Life (SNAMOPEQ), Polydisciplinary Faculty of Taza (FPT), Sidi Mohamed Ben Abdellah University (USMBA) [15].

### 2.3. Phytochemical Study

The collected leaves of *Chamaerops humilis* L. var. argentea Andre were dried and subjected to two types of extraction: aqueous extraction and organic extraction; the extraction procedure has been described in previous works of our laboratory [15, 27–30].

#### 2.3.1. Preparation of the Aqueous Extracts

Three aqueous extraction methods were applied: decoction, infusion, and maceration. The extraction by the three modalities was done separately. For each aqueous extraction modality, 10 g of *C. humilis* leaves was extracted with 100 mL of distilled water. After filtration, the solutions obtained were concentrated using a freeze-dryer (Heto PowerDry LL3000). The recovered residues were stored in amber glass vials at 4°C [15].

#### 2.3.2. Preparation of Organic Extracts

The organic extraction was carried out in two ways: hot with the soxhlet and cold by maceration with solvents of different polarities (ethanol, chloroform, and n-hexane). The organic extraction was performed separately for each solvent and modality used, in total 6 aqueous extracts were prepared (the ethanolic extract, the ethanolic macerated, the chloroformic extract, the chloroformic macerated, the hexanic extract, and the hexanic macerated). For each extraction, 40 g of plant material was used in a solvent volume of 400 mL. A rotary evaporator (Buchi R-210) was used at 40–50°C to remove the solvent and concentrate the organic extract into residues. These were stored in the dark at 4°C [15].

### 2.4. Cell Growth Inhibitory Activity of Aqueous and Organic Extracts of *Chamaerops humilis* L. var. argentea Andre: Phytotest *Lepidium sativum*

The phytotest *Lepidium sativum* is a biotest for the evaluation of antimitotic capacity based on the measurement of the length of the rootlet of a germinated seed of *Lepidium sativum* deposited in a medium containing the extract to be tested. In our study, we applied this test to evaluate the antimitotic capacity of aqueous and organic extracts prepared from the leaves of *C. humilis* following the method of [31]. To realize the test, 10 seeds of *Lepidium sativum* were germinated in petri dishes (55 mm) containing filter paper soaked with 1 mL of distilled water for 24 hours; then, 1 mL of the extract or reference standard to be tested was added at different concentrations to each dish, after which the dishes were incubated at 25°C. The results were read after 24 hours of incubation. For the reference drug, we used colchicine and the negative control was made by distilled water. During this test, we performed three replicates for each concentration tested. The percentage of cell growth inhibition was estimated by comparing the test batch with a control lot according to the formula below:

(1) $$\begin{array}{c} \%\text{of inhibition}={\frac{\text{LT}-\text{LC}}{\text{LT}}}^{*}100, \end{array}$$

where LT is the length of control rootlets and LC is the length of rootlets treated with the extract or the reference drug.

### 2.5. *In Vitro* Study of Antidiabetic Activity

#### 2.5.1. Inhibitory Activity of the Enzyme *α*-Amylase

The *α*-amylase inhibition test was performed using the procedure reported by [32], and the protocol followed is detailed in previous studies [15, 27, 29, 30, 33]. With a mixture containing 200 *μ*L of sample and 200 *μ*L of *α*-amylase enzyme (10 U/mL) prepared in 0.02 M sodium phosphate buffer (pH = 6.9), it was incubated for 10 min at 30°C. Subsequently, we added 200 *μ*L of the 1% starch solution to the reaction mixture. A second incubation was performed 3 min at 30°C. Then, we added 1 mL of the solution (DNS) and the reaction mixture was incubated again at 90°C for 10 min.

The reaction mixture was then diluted with 5 mL of distilled water. The absorbance value was measured at 540 nm by spectrophotometer (SPECUVIS2 UV/Vis, no.: HF1309003). Acarbose was used as a positive control. The percentage inhibition of *α*-amylase was calculated with the following formula:

(2) $$\begin{array}{c} \%\text{of inhibition}=\left[\frac{\left(\left({\text{Ac}}^{+}-{\text{Acb}}^{-}\right)-\left(\text{As}-\text{Ab}\right)\right)}{\left({\text{Ac}}^{+}-{\text{Acb}}^{-}\right)}\right]*100, \end{array}$$

where Ac^+^ is the absorbance of control with enzyme, Ac^−^ is the absorbance of control without enzyme, As is the absorbance of sample with enzyme, and Ab is the absorbance of sample without enzyme.

#### 2.5.2. Inhibitory Activity of the Enzyme *α*-Glucosidase

The inhibitory activity of aqueous and organic extracts of *C. humilis* leaves towards *α*-glucosidase was determined according to the protocol of Lordan and collaborators [34], detailed in our previous work [15, 27–30].

150 *μ*L of the sample at different concentrations was added to 100 *μ*L of *α*-glucosidase enzyme solution (0.1 U/mL) prepared in 0.1 M sodium phosphate buffer (pH = 6.7); the mixture was incubated at 37° C for 10 min. After this, we added 200 *μ*L of pNPG solution (1 mM). The reaction mixtures were incubated again at 37°C for 30 min. At the end, 1 mL Na_2_CO_3_ (0.1 M) was added to the reaction mixture. The absorbance was measured at 405 nm using a spectrophotometer (SPECUVIS2 UV/Vis, no.: HF1309003). The inhibitory capacity of *α*-glucosidase was expressed as percentage inhibition, and the median inhibitory concentrations (IC_50_) were calculated. Acarbose was used as a positive control.

#### 2.5.3. Inhibitory Activity of the Enzyme *β*-Galactosidase

The evaluation of the inhibitory power of *β*-galactosidase of aqueous and organic extracts from the leaves of *C. humilis* was carried out according to the method of [35], and the protocol was described in our previous work [15, 27, 29, 30, 33]; 150 *μ*L of different extracts or the reference drug was added to 100 *μ*L of *β*-galactosidase enzyme solution (1 U/mL) prepared in sodium phosphate buffer (0.1 M) at pH = 7.6. The mixture was incubated at 37°C for 10 min. Subsequently, a volume of 200 *μ*L of the substrate 2-nitrophenyl beta-D-galactopyranoside (1 mM) was added. The reaction mixture was incubated again at 37°C for 30 min. At the end of the protocol, we added 1 mL of Na_2_CO_3_ to stop the reaction and measured the absorbance at 410 nm using a spectrophotometer (SPECUVIS2 UV/Vis, no.: HF1309003). Quercetin was used as a positive control.

### 2.6. Acute Toxicity Assessment

Acute *in vivo* toxicity was performed on the decocted and ethanolic extract of *C. humilis* leaves. These extracts were chosen as they were found to be the most active *in vitro* among the other extracts. The acute oral toxicity test was performed according to the Organisation for Economic Cooperation and Development (OECD) guideline 423 [36].

#### 2.6.1. Animal Material

The *in vivo* toxicity study was performed on healthy, nulliparous, nonpregnant adult female Swiss mice weighing 25-30 g. The mice were provided by the animal facility of the Polydisciplinary Faculty of Taza, Sidi Mohamed Ben Abdellah University (USMBA) of Fez, Morocco. Mice were maintained, with free access to standard food and water, under standard conditions (12 h light/12 h dark at 23 ± 1°C). The mice were treated according to international guidelines for the care and use of animals in research [37].

#### 2.6.2. Acute Toxicity

The assessment of acute toxicity was carried out according to the recommendations of the Organisation for Economic Co-operation and Development guideline no. 423 [36]; the protocol followed has been described in detail in a previous work of our laboratory [38]. The decocted extract and the ethanolic extract of the leaves of *C. humilis* were tested at a dose of 2000 mg/kg with a volume of 0.5 mL/20 g body weight of the mouse. The experiment is carried out at each stage on three female Swiss mice for each product tested. This test was performed in two independent experiments in order to estimate the LD_50_. Therefore, 18 female mice were used. The first stage required a number of 9 mice for each stage which were fasted for a period of 4 h with free access to water; they were divided into 3 groups of three (3) mice each; the first and second groups were treated with the decocted and ethanolic extracts, respectively, and the last control group received distilled water. A behavioral observation was performed during the first 30 minutes and regularly during the first 24 hours after oral administration of the test products. According to the OECD guideline 423, the absence or the occurrence of substance-related mortality in a group dosed at a given stage specifies the next stage, either by stopping the experiment, administering the same dose to three more animals, or administering an immediately higher or lower dose to three more animals [36]. The mice were observed for a period of 14 days for changes in weight, mortality rate, animal behavior, and signs of toxicity. In addition, hydration and feeding were carried out on a daily basis.

### 2.7. Statistical Study and Principal Component Analysis (PCA)

GraphPad Prism 5 software was used to perform the statistical analysis of the data obtained using ANOVA variance followed by Tukey's test. When the *p* value is ≤0.05, the difference is considered statistically significant. Results are expressed as mean ± SEM.

For the correlation study between the content of total polyphenols, flavonoids, and catechic tannins in the aqueous and organic extracts determined in our previous work [15] and the results of the *Lepidium sativum* phytotest in the present study, we used Pearson's correlation analysis and principal component analysis (PCA) by Addinsoft XLSTAT software version 14.

## 3. Results

### 3.1. Cell Growth Inhibitory Activity of Aqueous and Organic Extracts of *C. humilis* Leaves: Phytotest *Lepidium sativum*

The results obtained on the inhibitory action of aqueous and organic extracts of *C. humilis* leaves on the cell growth of *Lepidium sativum* seeds are elucidated in the Figures 2–4.

From Figures 2 and 3, we notice that all aqueous and organic extracts have a cell growth inhibition capacity; this activity is proportional to the concentration tested. Firstly, the aqueous extracts expressed a maximum inhibitory effect at the concentration of 2 × 10^5^ *μ*g/mL: 75.76% for the decocted, 69.52% for the infused, and 75.93 for the macerated (Figure 2). Regarding the organic extracts at the concentration of 1.5 × 10^4^ *μ*g/mL; ethanolic extract and ethanolic macerated exerted a strong inhibition of cell growth with percentages of 89.86 and 90.68%, respectively, followed by chloroformic extract (71.15%), hexanic extract (65.32%), chloroformic macerated (61.57), and lastly hexanic macerated (59.57%) (Figure 3). In addition, colchicine also caused a high inhibition of 92.92% at the concentration 5 × 10^3^ *μ*g/mL (Figure 4).

In order to make a comparison between all the extracts tested, we calculated the IC_50_ of each extract and that of colchicine (Table 1).

The cell growth inhibitory action is higher for the organic extracts than for the aqueous extracts; indeed, the decocted and infused showed a higher inhibitory activity than the aqueous macerated with an IC_50_ of 9.624 × 10^3^ ± 95.97, 9.642 × 10^3^ ± 67.49, and 2.547 × 10^4^ ± 212.98 *μ*g/mL, respectively, with a nonsignificant statistical difference between the decocted and infused. Concerning the organic extracts, we found that ethanolic extract and ethanolic macerated expressed the highest values for the cell growth inhibition test with IC_50_ of 5.638 × 10^3^ ± 22.61 and 5.599 × 10^3^ ± 45.51 *μ*g/mL with a statistically insignificant difference, followed by chloroformic macerated (IC_50_ = 7.770 × 10^3^ ± 76.32 *μ*g/mL), hexanic macerated (IC_50_ = 9.599 × 10^3^ ± 69.90 *μ*g/mL), and chloroformic extract (IC_50_ = 1.054 × 10^4^ ± 93.12 *μ*g/mL). The analysis of variance showed a statistically insignificant difference between the hexanic extract and the hexanic macerated. In addition, colchicine showed a strong inhibitory activity expressed by the lowest IC_50_ (IC_50_ = 4.746 × 10^2^ ± 1.76 *μ*g/mL) with a statistically significant difference between all tested extracts.

### 3.2. *In Vitro* Study of Antidiabetic Activity

The study of the *in vitro* antidiabetic power of the aqueous and organic extracts prepared from the leaves of *C. humilis* was carried out by three tests for the inhibition of the enzymes *α*-amylase, *α*-glucosidase, and *β*-galactosidase. The expression of the results was done by calculating the IC_50_ (Table 2).

The tested aqueous and organic extracts showed an inhibitory activity of *α*-amylase with IC_50_ = 8.902 × 10^3^ ± 57.81 *μ*g/mL to 3.463 × 10^5^ ± 211.02 *μ*g/mL. For the aqueous extracts the decocted showed inhibitory activity: IC_50_ = 1.781 × 10^5^ ± 358.30 *μ*g/mL, followed, respectively, by the infused (IC_50_ = 2.579 × 10^5^ ± 690.80 *μ*g/mL) and the aqueous macerated (IC_50_ = 2.781 × 10^5^ ± 396.48 *μ*g/mL) with a statistically significant difference between the three extracts. Concerning the organic extracts, the ethanolic extract shows an inhibitory activity (IC_50_ = 8.902 × 10^3^ ± 57.81 *μ*g/mL), followed, respectively, by the chloroformic macerated (IC_50_ = 1.604 × 10^5^ ± 240.83 *μ*g/mL), the ethanolic macerated (IC_50_ = 1.754 × 10^5^ ± 107.08 *μ*g/mL) chloroformic extract (IC_50_ = 2.114 × 10^5^ ± 113.77 *μ*g/mL), hexanic extract (IC_50_ = 2.401 × 10^5^ ± 677.48 *μ*g/mL), and in the last place hexanic macerated extract (IC_50_ = 3.463 × 10^5^ ± 211.02 *μ*g/mL) with a statistically significant difference between all organic extracts. Acarbose shows high *α*-amylase inhibitory activity (IC_50_ = 6.160 10^2^ ± 5.00 *μ*g/mL). The evaluation of the inhibitory power of *α*-glucosidase *in vitro* shows that all the extracts present a remarkable inhibitory activity. Concerning the aqueous extracts, we found that the decocted has an inhibitory activity of IC_50_ = 2.540 × 10^2^ ± 3.14 *μ*g/mL followed by the infused (IC_50_ = 3.653 × 10^2^ ± 2.06 *μ*g/mL) with a statistically significant difference and the aqueous macerated comes last with a statistically nonsignificant difference with the infused (IC_50_ = 4.212 × 10^2^ ± 21.20 *μ*g/mL). Regarding the organic extracts, we found that ethanolic extract, ethanolic macerated extract, and chloroformic extract show relative IC_50_ inhibitory activity of 2.216 × 10^2^ ± 1.39, 2.352 × 10^2^ ± 1.13, and 2.804 × 10^2^ ± 0.75 *μ*g/mL, respectively; these three extracts show statistically insignificant difference between them. Chloroformic macerated recorded an *α*-glucosidase inhibition value equal to 4.293 × 10^2^ ± 2.65 *μ*g/mL, followed by hexanic extract (IC_50_ = 5.194 × 10^2^ ± 22.86 *μ*g/mL) and hexanic macerated (IC_50_ = 5.286 × 10^2^ ± 20.65 *μ*g/mL) with statistically nonsignificant difference between hexanic extract and hexanic macerated. Acarbose also showed high *α*-glucosidase inhibitory power (IC_50_ = 1.950 × 10^2^ ± 6.12 *μ*g/mL); the activity of acarbose is statistically insignificant with that of ethanolic extract and ethanolic macerated.

The aqueous and organic extracts also showed an inhibitory effect on *β*-galactosidase; for the aqueous extracts, the decocted recorded higher *β*-galactosidase inhibitory activity than the infused and aqueous macerated with IC_50_ values of 7.118 × 10^2^ ± 16.13, 9.050 × 10^2^ ± 9.33, and 8.544 × 10^2^ ± 13.66 *μ*g/mL, respectively. The analysis of variance (ANOVA) showed that there is a nonsignificant difference between the decocted and the other two aqueous extracts (infused and aqueous macerated). Regarding the organic extracts, ethanolic extract showed the most powerful inhibitory action (IC_50_ = 2.003 × 10^2^ ± 7.41 *μ*g/mL) followed by hexanic extract (IC_50_ = 2.593 × 10^2^ ± 19.13 *μ*g/mL), hexanic macerated (IC_50_ = 3.186 × 10^2^ ± 6.19 *μ*g/mL), chloroformic extract (IC_50_ = 3.598 × 10^2^ ± 7.29 *μ*g/mL), ethanolic macerated (IC_50_ = 4.792 × 10^2^ ± 13.43 *μ*g/mL), and chloroformic macerated (IC_50_ = 5.671 × 10^2^ ± 3.29 *μ*g/mL); analysis of variance revealed a nonsignificant difference between chloroformic extract and hexanolic macerated and between ethanolic extract and quercetin (IC_50_ = 1.711 × 10^2^ ± 5.00 *μ*g/mL).

### 3.3. Correlation Study between Chemical Composition and Cell Growth Inhibiting Effect of *C. humilis* Leaf Extracts

The correlation analysis between the chemical composition (total polyphenols, flavonoids, and catechic tannins) of the aqueous and organic extracts of *C. humilis* leaves and their antidiabetic and phytotoxic potencies was carried out on the basis of the results of the chemical content of the different extracts prepared in our previous work [15].

#### 3.3.1. Correlation Matrix

Principal component analysis (PCA) helped us to highlight possible correlations between the chemical content and the antidiabetic and phytotoxic activity of *C. humilis* leaves (Table 3).

#### 3.3.2. Graphical Representation of the Principal Component Analysis (PCA)

According to the PCA the two axes F1 and F2 present 86.73% of the total variance of the observations, which means that the interpretations will be highly significant, this analysis allowed us to define 3 groups (Figure 5):

- Group 1: consisting of ethanolic extract and ethanolic macerated which have high polyphenol contents and also express an antidiabetic effect for the enzymes *α*-amylase and *α*-glucosidase
- Group 2: includes chloroformic extract, chloroformic macerated extract, hexanic extract and hexanic macerated extract, which are rich in catechic tannins and flavonoids. These extracts show antidiabetic activity for the enzyme *β*-galactosidase and cytotoxic capacity via the phytotest *Lepidium sativum*
- Group 3: includes the aqueous extracts (decocted, infused, and macerated) which are characterized, according to this analysis, by a low chemical composition in total polyphenols, flavonoids, and catechic tannins; this group also presents low antidiabetic and antimitotic activities

### 3.4. Acute Toxicity

#### 3.4.1. Mortality and Signs of Acute Toxicity

Single-dose administration (2000 mg/kg) of the decocted and ethanolic extract did not cause any deaths in treated mice; however, a lack of appetite was observed on the first day of treatment. In addition, mice treated with ethanolic extract showed reduced mobility for 72 hours after treatment; however, mice from the control batch did not show any abnormal signs (Table 4).

#### 3.4.2. The Evolution of the Body Weight of Mice

The weight evolution of each animal was measured during the 14 days after the single administration of the two extracts: decocted and ethanolic extract; the weight of the groups treated with decocted and ethanolic extract showed no remarkable difference; however, the weight of the control group increased during the observation period with an average of 15.66% (Figure 6).

#### 3.4.3. Determination of the LD_50_

The determination of the LD_50_ was performed according to the OECD acute toxicity assessment method code no. 423; during the treatment period no deaths were observed, this indicates that the LD_50_ is greater than or equal to 5000 mg/kg. Furthermore, according to the Global System of Classification of Chemical Substances (GHS), both tested extracts belong to toxicity class 5 or not classified. Both extracts are thus considered to be mixtures with relatively low acute toxicity, but which may under certain conditions be hazardous to susceptible individuals [36].

## 4. Discussion

### 4.1. Phytotest *Lepidium sativum*

The *Lepidium sativum* test showed that the inhibitory effect on the growth of *Lepidium sativum* seed rootlets by the tested aqueous and organic extracts is dose dependent. Regarding the aqueous extracts, we found that the decocted and infused show better inhibitory activity presented by values of 9.624 × 10^3^ ± 95.97 and 9.642 × 10^3^ ± 67.49 *μ*g/mL, respectively, with a statistically nonsignificant difference. For the organic extracts, we found that the high *in vitro* antimitotic activity was presented by the ethanolic extract (IC_50_ = 5.638 × 10^3^ ± 22.61 *μ*g/mL) and the ethanolic macerated (IC_50_ = 5.599 × 10^3^ ± 45.51 *μ*g/mL) with a statistically nonsignificant difference between the two extracts. We can remark that the best results obtained via the *Lepidium sativum* phytotest are expressed by high polarity extracts prepared at high temperature (decocted, infused, and ethanolic extract) or by cold extraction by maceration with a long contact time between the plant material and the solvent (ethanolic macerated). This suggests that the active ingredients responsible for the antimitotic activity are better extracted with these extraction modalities. In addition, the cell growth inhibition or antimitotic effect could also be due to the chemical composition. Indeed, our recent study confirmed the richness of *C. humilis* leaves in total polyphenols, flavonoids, and catechic tannins [15]. Another study showed that the presence of phenolic compounds, alkaloids, and flavonoids are responsible for the antimitotic activity of the aqueous extract of *Ficus benghalensis* [39]. Studies conducted under the same operating conditions as ours found that both hamaline and harmalol alkaloids have high inhibitory activity on *Lepidium sativum* rootlet growth with an IC_50_ of 134.15 and 239.43 *μ*g/mL, respectively [40]. In addition, the methanolic extract and methanolic macerated of *Ajuga iva* had a strong antimitotic activity represented by an IC_50_ of 320.43 ± 8.96 and 375.77 ± 17.53 *μ*g/mL, respectively [38]. The antimitotic effect of *C. humilis* extracts could also be due to the mineral richness of the plant: iron (Fe): 82395.00, potassium (K): 9354.90, phosphorus (P): 1828.62, magnesium (Mg): 1312.47, sodium (Na): 627.03; copper (Cu): 542.64, calcium (Ca): 92.19, zinc (Zn): 66.15, selenium (Se): 3.00, and strontium (Sr):3.00 mg/kg) [15]. These mineral elements can be a means to fight or prevent the occurrence of cancer; several studies show that Zn deficiency leads to DNA oxidation and DNA breaks and chromosomal damage associated with increased cancer risk [41, 42]. Indeed, Zn plays a crucial role in DNA metabolism, and a deficiency in this element can induce important chromosomal mutations that increase the risk of cancer [43–45]. Selenium is another essential trace element that is vital for various cellular processes and is also frequently used to prevent the occurrence of cancer [46, 47]. In addition, both selenium and zinc play a role in the efficient progression of the DNA repair system, thereby mitigating DNA damage that could lead to cancer development [47, 48]. Magnesium (Mg) and potassium (K) may also play a protective role significantly against the development of colorectal cancer (CRC) [49, 50].

### 4.2. *In Vitro* Study of Antidiabetic Activity

The results of the *α*-amylase, *α*-glucosidase, and *β*-galactosidase enzymatic inhibition tests showed that all aqueous and organic extracts of *C. humilis* leaves show antidiabetic capacity *in vitro*. Firstly, the decocted showed a high inhibitory power for all three enzymes; this activity is higher than that of the infused and aqueous macerated, and this could be explained by the ability of the high temperature to extract better the molecules that have antihyperglycemic activity [15]. For the *α*-amylase and *β*-galactosidase enzymes, we found that ethanolic extract presented the best inhibitory activity compared to other organic extracts with IC_50_ = 8.902 × 10^3^ ± 57.81 and IC_50_ = 2.003 × 10^2^ ± 7.41 *μ*g/mL values, respectively. In addition, ethanolic extract and ethanolic macerated had remarkable *α*-glucosidase inhibitory power compared to other organic extracts presented by IC_50_ values of 2.216 × 10^2^ ± 1.39 and 2.352 × 10^2^ ± 1.13 *μ*g/mL, respectively, with statistically insignificant difference between them and with acarbose (1.950 × 10^2^ ± 6.12 *μ*g/mL). This suggests that polar solvent extraction at high temperature for 6-8 hours and maceration extraction for a longer period of 48 hours are capable of extracting the active ingredients responsible for this activity. These results can be explained by the results of the study of the chemical composition of the same extracts of the leaves of *Chamaerops humilis* [15], which showed that the ethanolic extract and the ethanolic macerated have high contents of total polyphenols of 96.99 ± 0.82 and 100.27 ± 0.66 *μ*g EAG/mE, respectively. Both of these extracts also showed a high content of flavonoids with values of 457.98 ± 5.18 and 468.25 ± 9.07 *μ*g TE/mgE, respectively, and of catechic tannins with 50.27 ± 0.99 and 52.11 *μ*g TE/mgE, respectively. ANOVA analysis proved that the statistical difference between ethanolic extract and ethanolic macerated is not significant [15]. Moreover, a recent study proved that polar extracts of *G. senegalensis* show better inhibitory activity on *α*-glucosidase [51]. The antihyperglycemic effect of all the extracts studied is also variable with respect to the three enzymes used which could be explained by the structural variation related to the origin of these enzymes [52]. The hypoglycemic effect of *Chamaerops humilis* could also be due to its mineralogical content; in our previous study, we found that the leaves of *C. humils* are rich in iron (82395.00 mg/kg), potassium (9354.90 mg/kg), phosphorus (1828.62 mg/kg), magnesium (1312.47 mg/kg), sodium (627.03 mg/kg), copper (542.64 mg/kg), calcium (92.19 mg/kg), and zinc (66.15 mg/kg) [15]. Firstly, potassium, zinc, and calcium play an important role in improving glucose tolerance and indirectly contribute in the management of type 2 diabetes; in addition, calcium also plays an important role in insulin release from islet *β*-cells [53, 54]. Mg supplementation may also be useful to resolve the phenomenon of insulin resistance [54, 55].

Our results are in agreement with an *in vivo* study conducted by Gaamoussi and collaborators, which demonstrated that plasma glucose levels in obese rats with hyperglycemia and hyperlipidemia decreased significantly with daily administration of *Chamaerops humilis* decocted from 12.04 ± 0.94 mmol/L to 6.10 ± 0.27 mmol/L after 15 days and to 4.84 ± 0.22 mmol/L after 30 days of treatment [22].

Studies conducted under the same experimental conditions in our laboratory on plants from the same region as our *Chamaerops humilis* plant found that the methanolic macerated of *Atractylis gummifera* recorded high inhibitory activity against the three enzymes *α*-amylase, *α*-glucosidase, and *β*-galactosidase with an IC_50_ of 557 ± 0.013, 743 ± 0.017, and 2443 ± 0.071 *μ*g/mL, respectively. Similarly, *Juglans regia* acetone macerated showed high inhibitory activity for *α*-amylase (IC_50_ = 5445.33 ± 82 : 58 *μ*g/mL), *α*-glucosidase (IC_50_ = 323 : 7 ± 1.71 *μ*g/mL), and *β*-galactosidase (IC_50_ = 811.2 ± 8.32 *μ*g/mL). *Ajuga iva* metanolic macerated showed a potent antidiabetic effect for *β*-galactosidase (IC_50_ = 146.47 ± 33.05 *μ*g/mL). The methanolic extract of *Haloxylon scoparium* also had a strong *α*-glucosidase inhibitory capacity (IC_50_ = 193.4 ± 8.57 *μ*g/mL) [28–30, 56].

### 4.3. Correlation between the Chemical Composition (Total Phenols, Total Flavonoids, and Catechic Tannins) and the Cell Growth Inhibitory and Antihyperglycemic Activity of Aqueous and Organic Extracts of *C. humilis* Leaves

According to the results of the principal component analysis (PCA), polyphenol content correlated well with antihyperglycemic activity for *α*-amylase (*r* = 0.6638) and moderately correlated with *α*-glucosidase (*r* = 0.5788) and *β*-galactosidase (*r* = 0.5712). In contrast, the inhibitory activity by *β*-galactosidase was better correlated with the content of catechic tannins (*r* = 0.7092) and flavonoids (*r* = 0.6345). According to these results, the hypoglycemic activity could be attributed to the active ingredients of different chemical nature, this activity could also be variable depending on the enzyme used. According to Sales and collaborators, the action of polyphenols and flavonoids in inhibiting *α*-amylase is explained by the formation of hydrogen bonds between its hydroxyl groups and the residues of the enzyme binding site [57]. The hypoglycemic effect of *Chamaerops humilis* leaves could also be due to the catechic tannins; according to Hosoyama and coworkers, tannins and ellagic acid derivatives from banaba (*Lagerstroemia speciosa* L.) are potent inhibitors of *α*-amylase [58]. In addition, a study indicated a strong correlation between phenolic compounds of *Gymnema montanum* leaves and the inhibitory effect of *α*-glucosidase and *α*-amylase activity *r*^2^ = 0.92 and *r*^2^ = 0.97, respectively [59].

Regarding the results obtained via the *Lepidium sativum* phyotest, a strong correlation was noticed between the *in vitro* antimitotic activity and the content of catechic tannins (*r* = 0.9370), flavonoids (*r* = 0.9153), and total polyphenols (*r* = 0.7612), which means that the *in vitro* cytotoxic activity might be due to several chemical families. This is in concordance with the study conducted by Zhao and collaborators who reported that phenolic compounds can influence hormone production and inhibit aromatase and therefore prevent cancer development [60]; flavonoids may also be effective in the cancer inhibition mechanism [61]. In addition, Stanisavljević and collaborators have shown strong correlations between the intensity of *in vitro* cytotoxic activity of *Pisum sativum* extracts and epigallocatechin and luteolin contents [62].

The present study clearly shows that *Chamaerops humilis* leaves possess both antimitotic and hypoglycemic effect; in the same sense, many studies have indicated the association between cancer and hyperglycemia; diabetes and insulin resistance could be the consequence of an as yet undiagnosed initial state of cancer; diabetes could also be related to the precancerous state of the pancreas which affects its insulin-secreting capacity [7]. Insulin resistance is associated with an inflammatory state that also promotes hepatic carcinogenesis. In addition, cancer is one of the most common causes of mortality in type 2 diabetes [11, 12]. According to Stocks and collaborators, for every 1 mmol/l increase in blood glucose, there is a 10-20% increase in cancer risk for both men and women [8]. Indeed, in the genesis of type 2 of diabetes, the existence of insulin sensitivity induces high blood levels of insulin and an increase in circulating levels of insulin-like growth factors (IGF). The IGFs stimulate cell proliferation in many organs, in particular the liver, pancreas, colon, ovary, and breast [7, 9, 10].

### 4.4. Acute Toxicity of *Chamaerops humilis* Leaves

During the observation period (14 days) following the administration of the decocted and the ethanolic extract at a dose of 2000 mg/kg, no deaths were recorded in the treated animals.

According to the method for determining the lethal dose (LD_50_) described by the European OECD guideline code no. 423, the tested extracts have a lethal dose (LD_50_) which is estimated to be ≥5000 mg/kg by the oral route. In addition, the Globally Harmonised System of Classification (GHS) allowed us to classify the decocted and the ethanolic extract in category V or unclassified [36], which means that these two extracts are considered to be a mixture with a proportionally low acute toxicity, but which may under certain conditions be hazardous to vulnerable persons [36].

During the observation period, we noted that mice treated with the decocted and ethanolic extract showed some clinical signs such as loss of appetite and reduced mobility during the first hours after administration. The mice returned to their normal state after 72 hours. However, the control group did not show any behavioral changes. These clinical signs could explain the weight evolution, which showed a slight decrease in body weight in the treated mice during the first 6 days and an increase in weight in the control group. A subacute toxicity study conducted in the rat animal model of *Haloxylon scoparium* decocted recorded a gain in body weight in rats treated with 500, 1000, and 2000 mg/kg. This growth was lower than that of the control group, 11.87%, 9.32%, and 8.59%, respectively, compared to the control group (18.67%) [63].

## 5. Conclusion

The present work focused on the search for new anticancer and antidiabetic agents via tests dedicated to the evaluation of the antimitotic and antihyperglycemic effects *in vitro* of three aqueous extracts and nine organic extracts of the leaves of *Chamaerops humilis* L. var. argentea Andre as well as the *in vivo* evaluation of the acute toxicity of the extracts which proved to be the most active *in vitro*, namely, that of the decocted and the ethanolic extract.

Our results show that all aqueous and organic extracts had antimitotic and antihyperglycemic effect *in vitro* with a variable degree with a better activity revealed mainly for ethanolic extract and ethanolic macerated for organic extracts and decocted for aqueous extracts. The mentioned extracts could constitute a natural source of anticancer and antidiabetic molecules for pharmaceutical applications.

The principal component analysis (PCA) showed that polyphenol content correlated better with antihyperglycemic activity for *α*-amylase (*r* = 0.6638). In addition, *α*-glucosidase inhibitory activity was better correlated with the content of catechic tannins (*r* = 0.7092) and with flavonoids (*r* = 0.6345). Concerning the *Lepidium sativum* phyotest, PCA showed that a strong correlation was observed between *in vitro* antimitotic activity and the content of catechic tannins (*r* = 0.9370), flavonoids (*r* = 0.9153), and total polyphenols (*r* = 0.7612). These results could lead to the conclusion that the antidiabetic activity and the antimitotic activity *in vitro* could be attributed to the active compounds that have different chemical natures.

Regarding the *in vivo* acute toxicity study, administration of a single dose of 2000 mg/kg of decocted and ethanolic extract did not cause any deaths; therefore, the LD_50_ is estimated to be ≥5000 mg/mL according to OECD and the tested extracts belong to class V or not classified according to the Globally Harmonised System of Classification (GHS).

## Figures and Tables

**Figure 1:** *Chamaerops humilis* L. var. argentea Andre (pictures taken in Bab Boudir, located 46 km from the city of Taza (North-East of Morocco). Geographical coordinates: N 34°24.904'', W 004°02.635'', Altitude: 1460 m).

**Figure 2:** Cell growth inhibitory activity of aqueous extracts of *C. humilis* leaves.

**Figure 3:** Cell growth inhibitory activity of organic extracts from *C. humilis* leaves.

**Figure 4:** Cell growth inhibitory activity of colchicine.

**Figure 5:** Principal component analysis (PCA) of the chemical composition and antidiabetic activity of aqueous and organic extracts of *C. humilis* leaves. D: decocted; I: infused; M.aq: aqueous macerated; E_t_OH: ethanolic extract; M.E_t_OH: ethanolic macerated; CHCl_3_: chloroformic extract; M.CHCl_3_: chloroformic macerated; Hex: hexanic extract; M.Hex: hexanic macerated; G1: group 1; G2: group 2; G3: group 3; TP: total polyphenols; TF: total flavonoids; CT: catechic tannins.

**Figure 6:** Weight evolution of the groups treated with decocted and ethanolic extract of *C. humilis* leaves and of the control group over 14 days.

**Table 1:** The median inhibitory concentrations (IC_50_) of the cell growth inhibitory effect of aqueous and organic extracts of *C. humilis* leaves.

Extracts	IC_50_ (*μ*g/mL)
Aqueous	
Decocted	9.624 × 10^3^ ± 95.97^a^
Infused	9.642 × 10^3^ ± 67.49^a,b^
Macerated	2.547 × 10^4^ ± 212.98^c^
Organics	
Ethanolic extract	5.638 × 10^3^ ± 22.61^d^
Ethanolic macerated	5.599 × 10^3^ ± 45.51^d^
Chloroformic extract	1.054 × 10^4^ ± 93.12^e^
Chloroformic macerated	7.770 × 10^3^ ± 76.32^f^
Hexanic extract	9.750 × 10^3^ ± 73.61^a,b,g^
Hexanic macerated	9.599 × 10^3^ ± 69.90^a,b,g^
Colchicine	4.746 × 10^2^ ± 1.76^h^

The results are expressed as the mean of three individual replicates (*n* = 3 ± SEM). Values with the same superscript letters in the same column are not significantly different (*p* < 0.05).

**Table 2:** Median inhibitory concentrations (IC_50_) in (*μ*g/mL) of *α*-amylase, *α*-glucosidase, and *β*-galactosidase inhibitory activity of aqueous and organic extracts of *C. humilis* leaves.

Extracts	*α*-Amylase	*α*-Glucosidase	*β*-Galactosidase
Decocted	1.781 × 10^5^ ± 358.30^a^	2.540 × 10^2^ ± 3.14^a^	7.118 × 10^2^ ± 16.13^a^
Infused	2.579 × 10^5^ ± 690.80^b^	3.653 × 10^2^ ± 2.06^b^	9.050 × 10^2^ ± 9.33^b^
Aqueous macerated	2.781 × 10^5^ ± 396.48^c^	4.212 × 10^2^ ± 21.20^b,c^	8.544 × 10^2^ ± 13.66^b^
Ethanolic extract	8.902 × 10^3^ ± 57.81^d^	2.216 × 10^2^ ± 1.39^a,d^	2.003 × 10^2^ ± 7.41^c^
Ethanolic macerated	1.754 × 10^5^ ± 107.08^e^	2.352 × 10^2^ ± 1.13^a,d^	4.792 × 10^2^ ± 13.43^d^
Chloroformic extract	2.114 × 10^5^ ± 113.77^f^	2.804 × 10^2^ ± 0.75^a,d^	3.598 × 10^2^ ± 7.29^e^
Chloroformic macerated	1.604 × 10^5^ ± 240.83^g^	4.293 × 10^2^ ± 2.65^c^	5.671 × 10^2^ ± 3.29^f^
Hexanic extract	2.401 × 10^5^ ± 677.48^h^	5.194 × 10^2^ ± 22.86^e^	2.593 × 10^2^ ± 19.13^g^
Hexanic macerated	3.463 × 10^5^ ± 211.02^i^	5.286 × 10^2^ ± 20.65^e^	3.186 × 10^2^ ± 6.19^e^
Acarbose	6.160 × 10^2^ ± 5.00^j^	1.950 × 10^2^ ± 6.12^d^	—
Quercetin	—	—	1.711 × 10^2^ ± 5.00^c^

The results are expressed as the mean of three individual replicates (*n* = 3 ± SEM). Values with the same superscript letters in the same column are not significantly different (*p* < 0.05).

**Table 3:** Correlation matrix between the chemical profile (total polyphenols, total flavonoids, and catechic tannins) and the antidiabetic antimitotic action of aqueous and organic extracts of *C. humilis* leaves.

Variables	Total polyphenols	Total flavonoids	Catechic tannins	*α*-Amylase	*α*-Glucosidase	*β*-Galactosidase	*Lepidium sativum* phytotest
Total polyphenols	1						
Total flavonoids	0.7556	1					
Catechic tannins	0.8924	0.9507	1				
*α*-Amylase	0.6638	0.4055	0.5189	1			
*α*-Glucosidase	0.5788	0.1613	0.3756	0.5970	1		
*β*-Galactosidase	0.5712	0.6345	0.7092	0.5363	0.0596	1	
*Lepidium sativum* Phytotest	0.7612	0.9153	0.9370	0.4456	0.1036	0.8592	1

**Table 4:** Mortality and clinical signs recorded in the acute toxicity study of ethanolic extract and decocted of *C. humilis* leaves.

	Ethanolic extract	Signs of acute toxicity	Decocted	Signs of acute toxicity	Control	Signs of acute toxicity
Step 1 (dose: 2000 mg/kg)						
Number of mice	3	(i) Anorexia (ii) Reduced mobility	3	(i) Anorexia (ii) Reduced mobility	3	—
Number of deaths	0		0		0	
Step 2 (dose: 2000 mg/kg)						
Number of mice	3	(i) Anorexia (ii) Reduced mobility	3	(i) Anorexia (ii) Reduced mobility	3	—
Number of deaths	0		0		0	

## Data Availability

The data generated or analyzed during this study are included in this article in form of tables and figures.

## Abbreviations

*C. humilis*: *Chamaerops humilis* L. var. argentea Andre
DNS: Dinitrosalicylic acid
pNPG: 4-p-Nitrophenyl-*α*-D-glucopyranoside
OECD: Organisation for Economic Co-operation and Development
PCA: Principal component analysis
IC_50_: The median inhibitory concentrations
GHS: Global system of classification of chemical substances
LD_50_: Lethal dose.
